This article has been retracted.

# Study of Deep Learning-Based Legal Judgment Prediction in Internet of Things Era

**DOI:** 10.1155/2022/8490760

**Published:** 2022-08-08

**Authors:** Min Zheng, Bo Liu, Le Sun

**Affiliations:** ^1^Hubei University of Science and Technology, Xianning, Hubei, China; ^2^Nanjing University of Information Science and Technology, Nanjing, China

## Abstract

Legal judgment prediction is the most typical application of artificial intelligence technology, especially natural language processing methods, in the judicial field. In a practical environment, the performance of algorithms is often restricted by the computing resource conditions due to the uneven computing performance of the devices. Reducing the computational resource consumption of the model and improving the inference speed can effectively reduce the deployment difficulty of the legal judgment prediction model. To improve the prediction accuracy, enhance the model inference speed, and reduce the model memory consumption, we propose a BERT knowledge distillation-based legal decision prediction model, called KD-BERT. To reduce the resource consumption in the model inference process, we use the BERT pretraining model with lower memory requirements to be the encoder. Then, the knowledge distillation strategy transfers the knowledge to the student model of the shallow transformer structure. Experiment results show that the proposed KD-BERT has the highest F1-score compared with traditional BERT models. Its inference speed is also much faster than the other BERT models.

## 1. Introduction

With the breakthroughs of deep learning-based natural language processing (NLP) algorithms [1], deep learning technology is widely used in various legal tasks. For example, automatic legal text generation and natural language case retrieval are both based on deep learning technology [2]. There is a very bright performance.

Legal judgment prediction is the most typical application of artificial intelligence technology, especially natural language processing methods, in the judicial field [3]. Legal judgment prediction tasks generally include subtasks such as crime prediction, relevant laws and regulations, and criminal sentence prediction. Through the study of legal materials, machine learning algorithms are used to build prediction models [4].

The practical application of the existing legal judgment prediction technology in the judicial field and its related products and solutions are gradually entering the public eye and being applied to assist the actual judicial process [5]. Legal judgment prediction technology is not intended to directly replace judges in adjudicating cases. But it is used to assist judges, provide reference for conviction, and improve judicial work efficiency. Although it cannot completely replace human judges, improving the accuracy of legal judgment prediction algorithms still has extremely high practical value and significance. The significance of legal judgment prediction is mainly reflected in the following two aspects [6].

For judges, the prediction of legal judgments can assist judges in adjudication and realize quick judgment of cases. For cases under trial, the legal judgment prediction algorithm can efficiently analyze the criminal behavior of the defendant in the case, and based on the learning of historical judgment data, recommend the relevant laws involved in the case, reason about the crime committed by the defendant, and give the judge more professional sentencing opinions. As judgment reference information, it can improve the work efficiency of legal professionals [7]. Through the combination of legal judgment prediction technology and judges, the speed of case processing can be improved, the case judgment process can be simplified, and the quick judgment of simple cases can be realized, so that legal workers can quickly handle simple cases and focus on handling complex cases.

For the parties, comprehensive intelligent guidance can be realized. A sound legal judgment prediction algorithm can provide corresponding legal guidance and assistance to people without legal background knowledge at a lower labor cost. Hiring a professional lawyer or knowing the legal knowledge on your own will have a certain capital or time cost for the parties who are not engaged in the legal related industry [8]. Through the legal judgment prediction algorithm, an intelligent litigation guidance system can be built, and by deeply mining judicial big data, a relatively complete information coverage of various crimes and laws can be constructed, providing professional case prediction and litigation guidance, and assisting the parties involved in litigation, or help litigation participants to make rational predictions.

To sum up, the application of legal judgment prediction is of great importance to the reform of the judicial field in the future [9]. A valuable supplement of legal advice provides corresponding legal guidance and assistance to people without legal background knowledge at a lower labor cost. Judicial adjudication assistance technology represented by legal judgment prediction is the main way to promote and realize judicial digitization, informatization, and intelligence. It can effectively solve many problems faced by current judicial practice and help to deepen the comprehensive supporting reform of the judicial system [10].

In a practical environment, the practicability of the algorithm is often restricted by the computing resource conditions due to the uneven computing performance of the devices that deploy the prediction algorithm [11]. Reducing the computational resource consumption of the model and improving the inference speed can effectively reduce the deployment difficulty of the legal judgment prediction model, enhance its practical value, provide efficient, convenient, and accurate services for judges and parties, and promote the development of judicial intelligence [12].

The pretraining model represented by BERT performs well in various natural language processing tasks [2]. However, due to the use of a deep transformer encoder, the pretraining model generally has many parameters, and the pretraining model needs to occupy a high memory in fine-tuning and inference. Although the additional computational overhead caused by building independent models for multiple subtasks is avoided through joint training and parameter sharing, the actual model inference speed is still slow. The BERT-based pretraining model based on the 14-layer transformer structure and BERT-Text-CNN has more than 115M encoder parameters, which seriously hinders the application of decision prediction algorithms based on pretrained models in practices with limited computing resources [13].

To improve the model inference speed, the model memory consumption is reduced and the practicability of the model without losing the performance of the model is enhanced, we propose a BERT knowledge distillation-based legal decision prediction model, called KD-BERT. The main contributions are as follows:

1. The BERT pretraining model with lower memory requirements is used as an encoder to reduce resource consumption in the model inference process.
2. Using the knowledge distillation strategy and the BERT knowledge distillation strategy, the knowledge information in the teacher model is transferred to the student model of the shallow transformer structure through knowledge distillation.
3. A knowledge distillation strategy that incorporates teacher model evaluation is proposed. The performance of the teacher model in the training data is used as the basis for the student model to learn from the teacher model and the label data. Dynamic weights are used to balance the label loss and distillation loss to obtain student models.

The rest of the structure is as follows: Section 2 introduces related work, Section 3 introduces the method of BERT knowledge distillation-based legal decision prediction, Section 4 shows the experiments, and Section 5 concludes this paper.

## 2. Related Work

Work [14] builds the first Legal Judgment Prediction (LJP) model for UK court cases by creating a labeled dataset of UK court decisions and subsequently applying the machine learning model with high performance and experimentally demonstrating the high performance capabilities of the proposed LJP model. Work [15] presents a multitask Legal Judgment Prediction model that combines the subtask of allegation severity with the defendant's position, enabling it to focus on contextual information about the defendant. Experiments show that the model achieves better performance on the public CAIL2018 dataset. Work [16] proposes a controlled tensor-based decomposition algorithm, TenLa, for computer-aided adjudication. First, the legal case is represented as a three-dimensional tensor, then a new tensor decomposition algorithm is proposed, and finally the kernel tensor obtained by ConTen is used to train OLASS. Work [17] analyses machine learning models to assist in determining the outcome of preliminary cases and applies machine learning models to predict the likely application of the IPC part of the case. The experimental results show that the machine learning model predictions can help judges and lawyers to make decisions as well as nonlegal professionals to decide the cases.

Work [18] finds accuracy by using a support vector machine (SVM) algorithm to solve the large number of cases remaining in the Indian judicial system each year, with a focus on “dowry death” related cases, predicting justice based on the analysis of judicial arguments to achieve justice. Work [19] uses transformers' bidirectional encoder (BERT), applied to Legal Judgment Prediction and violation prediction. It investigates how to handle long legally relevant documents and the importance of pretraining documents in the domain of the target task. The research [20] reviews the challenges faced by judgment prediction systems using deep learning model cases and also reviews current codec architectures with attention mechanisms for transformer model prediction systems for legal judgment and reviews the existing hierarchical attentional neural network models used in legal verdict prediction systems.

Work [21] uses convolutional neural networks (CNNs) to solve the problem of predicting the European Court of Human Rights (ECHR) judgments automatically by pretraining and customizing the textual representations considering word embeddings and statistically testing them to gather sufficient statistical evidence. Work [22] applies supervised machine learning model to cases about the “domestic violence for women” and proposes a model for predicting the guilt of the accused. Experiments have shown that the performance and accuracy of legal prediction systems can reduce the workload of legal professionals. In work [23], the authors proposed an attentional neural network, Legalat, and used the relevant literature to improve the performance and enhance the interpretability of the charge prediction task to achieve matching the facts of the case to the relevant law, with the final verdict being rendered according to the relevant legal provisions, and finally achieving optimal performance on the actual dataset.

Work [24] proposed a process supervision-based model for predicting legal decisions. Work [25] proposed an evaluation model of court judgment system based on grey system theory and BP neural network algorithm. Work [26] proposed a decision assistance method using restricted tensor factorization and relation-driven recurrent neural networks. Work [27] proposed a legal text recognition model based on conditional random fields and bidirectional Long Short-Term memory networks.

## 3. BERT Knowledge Distillation-Based Legal Decision Prediction

In natural language processing area, using a pretraining model with a huge amount of data can effectively improve the performance of the model in the target task. However, the huge number of parameters of the pretraining model also makes it difficult to directly apply it to online tasks. Using knowledge distillation for the pretraining model can effectively improve the practicability of the model.

The purpose of knowledge distillation is to achieve knowledge transfer between models by letting the untrained student model learn the trained teacher model. Generally, the structure of the student model is simpler than that of the teacher model, and it has fewer layers or parameters. Through knowledge distillation, the student model can obtain similar performance to the teacher model, accelerate the model inference, and reduce the memory usage of the model. The structure of knowledge distillation is shown in Figure 1.

As shown in the figure, knowledge distillation generally uses the output layer distribution of the teacher model as a soft label, and the labels in the dataset as hard labels. Imitation of the teacher model. In order to further narrow the gap between the teacher model and the student model, the intermediate layer distribution loss of the teacher model and the student model can also be added in the distillation process. The loss function *L* of knowledge distillation can be expressed as follows:

(1) $$\begin{array}{c} L=\mu L_{qa}+\pi L_{1}+\rho L_{2}. \end{array}$$

Among them, *L*_*qa*_, *L*_1_, and *L*_2_ represent the distillation loss from the soft label, the supervision loss from the dataset label, and the intermediate layer distribution loss of the teacher model and the student model, respectively, and *μ*, *π*, and *ρ* represent the weights of each loss function.

On the premise of ensuring the performance, we try to use the knowledge distillation strategy. The BERT model is used as the teacher model for knowledge distillation to reduce the redundant parameters and enhance the inference speed.

Referring to the existing research, we tried to use two mainstream knowledge distillation strategies for pretraining models: knowledge distillation and BERT knowledge distillation strategy to compress the model and combined the characteristics of legal judgment prediction to further improve the predicition accuracy.

### 3.1. Knowledge Distillation Strategy

Knowledge distillation is a knowledge distillation strategy to alleviate the lack of resources in large-scale model training for pretraining models such as BERT, which can compress the original BERT pretraining model into an equally effective lightweight shallow student model of the layer network.

Different from the traditional knowledge distillation strategy that only uses the output of the last layer of the teacher network for refining, the patient knowledge distillation strategy introduces an additional intermediate layer distribution loss to make full use of the rich information in the deep structure of the teacher network.

(2) $$\begin{array}{c} L_{qs}=\sum_{i=1}^{M}\sum_{k=1}^{K}\left\|\frac{h_{i,k}^{s}}{{\left\|k\right\|}_{2}}-\frac{h_{i,I_{qs}\left(k\right)}^{u}}{{\left\|h_{i,I_{qs}\left(k\right)}^{u}\right\|}_{2}}\right\|, \end{array}$$

where *M* represents the number of layers in the student network, *K* represents the number of training samples, and *h*_*i*,*k*_^*s*^ and *h*_*i*,*I*_*qs*_(*k*)_^*u*^  represent the representations of the corresponding vectors of the teacher model and the student model at the corresponding hidden layer positions.

The student model is initialized with the first few layers of the teacher model and distributing the loss through the middle layers in training, we patiently learn the vector representations at character positions from multiple middle layers of the teacher model to gradually extract knowledge.

Experiments demonstrate that the distillation schemes can exploit much information in the hidden layers of the teacher and approve the student model to learn the teacher by using the multilayer distillation process.

The patient knowledge distillation strategy can effectively compress the BERT teacher model with a 15–28-layer transformer structure into a student model with a 2–5-layer transformer structure, which significantly improves the training and prediction efficiency without sacrificing the accuracy of the model.

### 3.2. Small KD-BERT Knowledge Distillation Strategy

Small KD-BERT is a knowledge distillation strategy specially designed for transformer-based models. With this new knowledge distillation strategy, the large amount of knowledge encoded in the large BERT pretrained model can be well transferred to the small KD-BERT student model.

The small KD-BERT student model itself is a shallow transformer model with a low hidden layer dimension. In addition to accepting the soft label loss of the output distribution and the supervised label loss, by encouraging the small KD-BERT student model to imitate the word embedding layer output, hidden layer output, and attention matrix of the BERT teacher model, it is trained to obtain close performance to the teacher model, where, because the dimensions of the embedded layer and hidden layer of the small KD-BERT student model and the teacher model are different, a method similar to the embedding layer factorization in BERT is used to match the hidden layer of the teacher model and the student model through mapping.

The distillation loss of the K-layer small KD-BERT student model can be expressed as follows:

(3) $$\begin{array}{c} J_{\text{an}}=\frac{1}{k}\sum_{i=1}^{k}\text{MSE}\left(F_{i}^{s},F_{i}^{T}\right),\\ J_{\text{hd}}=\text{MSE}\left(L^{S}M_{k},L^{T}\right),\\ J_{\text{ed}}=\text{MSE}\left(R^{S}M_{e},R^{T}\right),\\ J_{DS}=-\text{softmax}\left(a^{T}\right)\cdot \text{log}\left(\text{tan}h\left(\frac{a^{T}}{T}\right)\right),\\ J_{ly}\left(S_{n},T_{q\left(n\right)}\right)=\left\{\begin{array}{cc} J_{\text{ed}}\left(S_{0},T_{0}\right), & n=0,\\ J_{\text{hd}}\left(Sm,T_{g\left(m\right)}\right)+L_{\text{an}}\left(Sm,T_{g\left(m\right)}\right), & Nn0,\\ J_{\text{DS}}\left(S_{\left(N+1\right)},T_{\left(N+1\right)}\right), & n=\left(N+1\right). \end{array}\right.\;\; \end{array}$$

Among them, *F*  is the attention matrix, *L* is the hidden layer output, *R* is the embedding layer output, and *M* is the mapping matrix.

Empirical research results show that small KD-BERT is effective, achieving results close to BERT on the GLUE benchmark, 8 times smaller in size, and 10 times faster than BERT in inference.

In addition, compared with the patient knowledge distillation strategy, the transformer structure in small KD-BERT can have a different hidden layer dimension from the teacher model. The structure design of the student model small KD-BERT is more flexible, the number of parameters of the student model can be further reduced, and the inference speed is further improved.

## 4. Experiment

### 4.1. Experimental Parameter Settings

In the tasks of crime prediction, relevant law recommendation, and sentence prediction tasks, ALBERT knowledge distillation uses the same Adam optimizer as BERT_14_ for training, and the learning rate is set to 0.01. In knowledge distillation, the distillation temperature parameter *T* is set to 3, and the student model BERT1 and BERT2 uses the Adam optimizer for training, and the learning rate is set to 0.001. The text length is limited to 256 words, and the batch size is set to 64. Limited by video memory, the gradient accumulation method is adopted, the actual batch sizes of BERT14, BERT1, and BERT2 are 18, 36, and 128, respectively, and the gradient is updated once every accumulation to 256.

In knowledge distillation, all CAIL20202 data is used as augmented data. For augmented data, only nonlabeled losses such as distillation loss and intermediate layer distribution loss are calculated, and labeled training is not performed based on augmented data. BERT14, BERT1, and BERT2 are trained on the training set for 100 rounds, and each round is verified twice on the validation set, and the model with the best verification result is tested on the test set. Each model directly predicts the task of crime prediction and legal article recommendation. For the sentence prediction task, a step-by-step prediction strategy, called sentence fine-grained prediction, is developed. The sentence prediction task builds a word-word mixture based on TextCNN on the basis of each model. Embedding model uses GBM model for fine-grained sentence prediction task for training, and other parameter settings are consistent with BERT14.

### 4.2. Experimental Results

The evaluation indicators of BERT14, BERT1, and BERT2 in the subtasks of crime prediction, relevant laws and regulations, and crime and sentence prediction are F1, R-F1, and accuracy. The performance of each model is shown in Table 1.

As can be seen from Table 1, the overall performance of the BERT14 model is closest to that of BERT1. Using the BERT pretraining model as the encoder pretraining model will not have a big influence on the model performance. Through small KD-BERT and the patient knowledge distillation strategy, it can enable the student model to effectively learn to imitate the performance of the teacher model, and the student model based on the small KD-BERT strategy has certain advantages over the student model based on the patient knowledge distillation strategy. Student model performance is degraded due to the teacher model bias.

To compare the difference in the inference speed between the student model and the teacher model, BERT14, BERT1, and BERT2 were used to infer the same 800 cases of data one by one. The average single data inference time, BERT14, BERT1, and BERT2 inference speed comparison is shown in Table 2.

As can be seen from Table 2, although BERT14 uses the hidden layer cyclic calculation to effectively compress the model volume, BERT14 cannot effectively improve the calculation efficiency because it does not actually reduce the calculation amount. The volume of BERT2 after knowledge distillation is about 58% of that of BERT14, the inference speed is increased by about 1.2 times. The volume of BERT1 is about 15% of the volume of the BERT14 model, and the inference speed is increased by about 7 times.

## 5. Conclusion

To improve the prediction accuracy, enhance the model inference speed, and reduce the model memory consumption, we proposed a BERT knowledge distillation-based legal decision prediction model, called KD-BERT. We used the BERT pretraining model with low memory requirements to be the encoder to reduce the resource consumption in the model inference process. Then, the knowledge distillation strategy transfers the knowledge to the student model of the shallow transformer structure. Experiment results show that the proposed KD-BERT has the highest F1-score than that of traditional BERT models. Its inference speed is also much faster than that of other BERT models.

## Figures and Tables

**Figure 1:** Process of KD-BERT.

**Table 1:** Performance comparison between KD-BERT and various knowledge distillation models.

Model	Layers# of encoders	Model parameters (M)	F1	R–F1	ACC1	ACC2
BERT14	14	115	0.892	0.844	57.5	77.2
BERT1	3	80	0.898	0.810	56.3	75.4
BERT2	6	28	0.884	0.832	56.8	75.7
Small KD-BERT	3	15	0.892	0.845	56.1	75.8
KD-BERT	4	13	0.912	0.887	59.2	79.6

**Table 2:** Comparison of inference time between KD-BERT and various knowledge distillation models.

Model	Encoder layers	Model size (M)	Model ratio	Average time (s)	Average speed
BERT14	14	115	1.2x	0.052	1.2x
BERT1	4	30	0.28x	0.044	1.1x
BERT2	6	80	0.62x	0.028	1.9x
**KD-BERT**	**4**	**15**	**0.09x**	**0.0006**	**7.68x**

## Data Availability

The labeled datasets used to support the findings of this study are available from the corresponding author upon request.
